# Electroacupuncture Regulates TRPV1 through PAR2/PKC Pathway to Alleviate Visceral Hypersensitivity in FD Rats

**DOI:** 10.1155/2021/1975228

**Published:** 2021-11-29

**Authors:** Yong-li Han, Xing-ming Peng, Hong-xing Zhang, Song Chen, Liang-yu Zhang

**Affiliations:** ^1^College of Acupuncture and Orthopedics, Hubei University of Chinese Medicine, Wuhan, Hubei 430061, China; ^2^Institute of Internal Medicine, Huangjiahu Hospital of Hubei University of Chinese Medicine, Wuhan, Hubei 430065, China; ^3^Department of Acumoxa, Wuhan Intergrated TCM & Western Medicine Hospital, Wuhan, Hubei 430022, China; ^4^Second People's Hospital of Jingzhou, Jingzhou, Hubei 434099, China; ^5^Digestive Endoscopy Treatment Center, Second Affiliated Hospital, Nanjing University of Chinese Medicine, Nanjing, Jiangsu 210017, China

## Abstract

Visceral hypersensitivity (VH) is the predominant pathogenesis of functional dyspepsia (FD). Duodenal hypersensitivity along with nausea further reduces the comfort level in gastric balloon dilatation and inhibits gastric receptive relaxation. The potential mechanism behind electroacupuncture- (EA-) mediated alleviation of VH has not been elucidated. In an FD rat model with tail clamping stress, iodine acetamide (IA) induced VH. The rats were treated with EA with or without PAR2 antagonist FSLLRY-NH2, and the body weight, gastric sensitivity, compliance, and gastrointestinal motility were determined. Mast cells and activated degranulation were stained with toluidine blue (TB) staining and visualized under a transmission electron microscope (TEM). Immunofluorescence was used to detect the expression of PAR2, PKC, and TRPV1 in the duodenum and dorsal root ganglion (DRG) and that of CGRP, SP in DRG, and c-fos in the spinal cord. EA alone and EA + antagonist enhanced the gastrointestinal motility but diminished the expression of TRPV1, CGRP, SP, and c-fos-downstream of PAR2/PKC pathway and alleviated VH in FD rats. However, there was no obvious superposition effect between the antagonists and EA + antagonists. The effect of EA alone was better than that of antagonists and EA + antagonists 2 alone. EA-induced amelioration of VH in FD rats was mediated by TRPV1 regulation through PAR2/PKC pathway. This protective mechanism involved several pathways and included several targets.

## 1. Introduction

Functional dyspepsia (FD), a common chronic gastrointestinal disease, is characterized by upper abdominal pain or burning sensation, postprandial fullness, early satiety, belching, and other symptoms [1]. According to the diagnostic criteria of Rome IV functional gastrointestinal diseases, FD was classified into two subgroups: epigastric pain syndrome (EPS) and postprandial distress syndrome (PDS) [2]. The global prevalence rate of FD is 21.8%, though there is a significant variation of this rate from country to country [3]. Although the pathophysiological mechanism of FD remains unknown to date, its association with brain–intestinal interaction, gastrointestinal motility, visceral hypersensitivity (VH), gastrointestinal microbiota, mucosal barrier, and immune activation, and abnormality of the central nervous system, resulting from the comprehensive action of multiple factors, has been investigated [4].

Along with EPS symptoms, VH is also associated with nonpainful sensations (such as postprandial fullness, abdominal distension, and hiccups) [5]. Moreover, an increase in gastrointestinal sensitivity gradually intensifies the severity of gastrointestinal symptoms in patients suffering from FD. Research in Malaysia confirmed the onset of FD resulting from a high intake of chili peppers [6]. Selectively activated by capsaicin, transient receptor potential vanilloid-1 (TRPV1) induces the release of neuropeptides, including calcitonin gene-related peptide (CGRP) and P substance (SP). These neuropeptides increase VH and induce FD symptoms (including abdominal pain and nausea) [7]. Various stimuli result in the activation and degranulation of mast cells, releasing a large amount of trypsin and tryptase (TRY), which, in turn, activate protease-activated receptor 2 (PAR2) on nociceptive neurons, causing neuronal excitement and releasing nociceptive neurotransmitters CGRP and SP, ultimately increasing VH in patients with FD [8]. PAR2 and TRPV1 are colocalized in the primary afferent nerve and coexpressed in more than 60% of L4–6 DRG cells, whereas both CGRP and SP are evident in 20% of the 35% PAR2-expressing neurons [9]. A synergistic effect of PAR2 with TRPV1 on VH regulation is documented. Excessive activation of the PAR2-PKC pathway mediates TRPV1 phosphorylation and decreases the TRPV1 opening threshold and abnormal visceral pain perception, eventually leading to VH [10, 11].

Acupuncture has been explored as a potentially effective nondrug therapy for functional gastrointestinal diseases. Efficacy of the electroacupuncture (EA) therapy in improving the dyspeptic symptoms of refractory FD patients was confirmed in a Chinese randomized controlled trial (RCT) involving 200 refractory FD patients, and its effect was found to be better than that of the sham acupuncture group [12]. High-quality RCT also validated significant amendment with acupuncture thrice a week in the PDS symptoms of FD patients with improved quality of life. After termination of the treatment, the curative effect was maintained for 12 weeks, and the adverse reactions were minimal during the treatment period [13]. Our previous studies also reported that EA at the acupoints (“Zusanli” and “Taichong”) improved gastrointestinal motility and reduced low-grade duodenal inflammation in FD model rats [14, 15], substantiating the effectiveness of these two acupoints. The present study employed iodine acetamide (IA) combined with tail clamping stress to induce the FD rat model and explored the effect of EA on intestinal hypersensitivity in FD rats to determine whether EA alleviated intestinal hypersensitivity through the PAR2/TRPV1 signal pathway.

## 2. Materials and Methods

### 2.1. Animal

The Experimental Animal Center of the Three Gorges University (license number is SCXK (E) 2017–0012) provided 42 SPF male 10-day-old SD (Sprague-Dawley) young rats. The animals were maintained in the Experimental Center of traditional Chinese Medicine of Hubei University of Traditional Chinese Medicine. The animal feeding environment was as follows: room temperature (20 ± 2)°C, humidity (50 ± 10)%, normal light replacement, 24 h supply of aseptic feed, and drinking water. All animals were fed adaptively for three days before the initiation of the experiment.

### 2.2. Construction and Evaluation of FD Model

Studies have shown that iodoacetamide intragastric administration can simulate better the pathological states of human visceral hypersensitivity and reduce gastric compliance [16, 17]. In contrast, the traditional tail pinch stress method simulates the symptoms of reduced food intake, delayed gastric emptying, and increased visceral sensitivity, which also stimulates rats to produce emotional changes such as anxiety and irritability, and simulates some causes of FD to a certain extent [18]. In order to completely simulate the symptoms and pathological states of FD patients, such as high visceral sensitivity, reduced gastric compliance, and delayed gastric emptying, the FD rat model was induced by IA along with tail clamping stress. The 42 10-day-old SD rats were randomly divided into control group (*n* = 8) and model group (*n* = 34). Each rat in the control group was administered 2% sucrose solution 0.2 mL/d for six days, and each rat in the model group was given a mixture of 0.1% IA and 2% sucrose 0.2 mL/d for six days. Following intragastric administration, the rats in each group were fed normally to the age of seven weeks. From the age of seven weeks, the rats in the model group were induced by Guo's tail stimulation method for one week; however, the control group did not receive any intervention until the rats were eight weeks old. The body weight of rats was recorded during intragastric administration (from 13 days to 20 days old). At the age of eight weeks, the gastric sensitivity of rats was estimated (the rate of EMG root mean square change of cervical trapezius muscle during gastric dilatation stimulation reflected the evaluation index), and compliance was evaluated (the volume/pressure of intragastric balloon during gastric dilatation stimulation represented the evaluation index). According to the evaluation of the model, 32 rats in the model group were successfully established.

### 2.3. Animal Grouping and Intervention

Thirty-two rats were randomly classified into four groups, with eight rats in each group (two cages/group; four rats/cage). Overall, there were five groups: control group, model group, EA group, antagonist group, and EA + antagonist group. The control group and model group did not receive any intervention for 14 consecutive days. EA group had acupuncture on both sides of “Zusanli” (located at about 5 mm under the fibula head under the knee joint of rats) and “Taichong” (located at the depressions between the first and second metatarsals of the dorsal foot of the left hindlimb) with one-off acupuncture of 0.30 mm × 25 mm specification, direct needling 1 mm, and Han's acupoint nerve stimulator with the continuous wave, frequency 2 Hz, current intensity 1 mA. The degree implied no obvious discomfort and rejection in the limbs of the rats. The needle was retained for 30 min, once daily for 14 days. The antagonist group [19] received no intervention in the first 11 days, until the intrathecal injection of 10 *µ*L PAR2 antagonist FSLLRY-NH2 (10 mg/L) was continuously given three days before sampling once daily three times. The EA + antagonist group had the previously mentioned EA intervention for 14 days, and intrathecal injection of FSLLRY-NH2 was given three days before sampling.

### 2.4. Organizational Preparation

After completing all interventions, the rats were fasted for 24 h and weighed and were fed 2 mL/100 g nutritious semisolid paste (5 g carboxymethylcellulose, 8 g milk powder, 4 g white sugar, and 4 g starch dissolved in 125 mL distilled water to prepare 150 g nutritious semisolid paste) and 1 mL/100 g ink according to their body weight. Following intragastric administration for 1 h, the rats were killed by cervical dislocation. The stomach and small intestine were collected, and the stomach's total weight and net weight were recorded. The difference between the two was calculated as the gastric residual weight, and then, the gastric residual rate was calculated as follows: (total gastric weight-Wei net weight)/given paste weight × 100%. The total length of the small intestine and the propulsive length of the ink (that is, the length from the pylorus to the front of the ink) were measured. Furthermore, the tissues of the gastric antrum, duodenum, T8–10 spinal cord, and dorsal root ganglion were frozen in liquid nitrogen and preserved in 4% paraformaldehyde and 2.5% glutaraldehyde fixation solution, respectively.

### 2.5. Hematoxylin-Eosin (HE) Staining

After dewaxing the paraffin sections of the stomach and duodenum to water, these sections were stained with hematoxylin staining solution, dehydrated, then placed in eosin dye solution for 5 min, then again dehydrated and sealed, and examined by the microscope, and the images were collected for analysis. The nucleus was stained blue and the cytoplasm red.

### 2.6. Toluidine Blue (TB) Staining

The paraffin sections of duodenal tissue were dewaxed to water, stained with TB dye for 2 min, and differentiated with 0.5% glacial acetic acid until the nuclei and particles were visible. After drying for more than 4 h, the sections were placed in xylene to make them transparent and sealed with neutral gum. The cytoplasm of mast cells was purplish-red, and mast cells were counted under the microscope.

### 2.7. Transmission Electron Microscope (TEM)

After rinsing, the duodenal tissue was fixed by 1% osmic acid 0.1 m phosphate buffer (pH 7.4) at room temperature (20°C) for 2 h, dehydrated by a series of alcohol gradients, and then permeated with acetone: epoxy resin (2 : 1), acetone: epoxy resin (1 : 1), epoxy resin, each time for 8–12 h. The infiltrated duodenal tissue was embedded in epoxy resin and then sliced and stained with uranium and lead. Finally, the ultrastructural characteristics of fragmentary or allergic degranulation of duodenal mast cells were visualized under the electron microscope.

### 2.8. Immunohistochemistry

Paraffin sections of duodenal tissue were dewaxed to water and placed in a repair box filled with EDTA antigen repair buffer (pH 9.0) for antigen repair. The slices were shaken dry. A circle around the tissue was drawn with a histochemical pen, and then, the slices were incubated with BSA dripping in the circle for 30 min. After dripping an anti-(TRY), washing the slide on the slice, and drying it, the covering tissue of the second antibody (HRP labeled goat anti-rabbit) was added to the circle and incubated for 50 min at room temperature. After washing the slide again and shaking it dry, DAB chromogenic agent was added to the circle, dehydrated with anhydrous ethanol, and sealed with xylene transparent neutral gum. In mast cells, TRY was mainly expressed in the granules in the cytoplasm, which was stained brown and yellow. Each slice in each group was randomly screened with at least three 200-fold visual fields to be photographed. While taking photos, the whole field of vision of the organization should be filled to ensure consistency in the background light of each photo. The same brown and yellow color was selected as the unified standard for judging the positivity of all photos by using Image-Pro Plus 6.0. The integrated optical density (IOD) of each positive photo was obtained by analyzing each photo.

### 2.9. Immunofluorescence

Paraffin sections of duodenal tissue were dewaxed to water sections and placed in a repair box filled with EDTA antigen repair buffer (pH 9.0) for antigen repair. The slices were shaken dry, incubated for 30 min with BSA dripping in the circle after drawing a circle around the tissue with a histochemical pen. The first antibody (including PAR2, PKC, and TRPV1) was added to the slice. After washing and drying the slide, the second antibody (including CY3-labeled goat anti-mouse and CY3-labeled goat anti-rabbit) covering tissue of the corresponding species was introduced in the circle and incubated for 50 min at room temperature. After washing the slide again and shaking it dry, DAB chromogenic agent was added to the circle, dehydrated with anhydrous ethanol, and sealed with xylene transparent neutral gum. The images were observed and collected under the fluorescence microscope. The nucleus stained by DAPI was blue under UV excitation, whereas the positive expression was red or green light labeled with the corresponding fluorescein. The same method was adopted to detect the expression of PAR2, PKC, TRPV1, CGRP, SP in DRG, and c-fos in the spinal cord. Each slice in each group was randomly selected with at least three 200-fold visual fields to be photographed. The red fluorescent monochromatic photos were converted into black-and-white pictures with the help of the Image-Pro Plus 6.0 software. The same black was then selected as the unified standard to judge the positive of all photos. Each photo was analyzed to retrieve the individual IOD value.

### 2.10. Western Blot

Add tissue protein extraction reagent 10 times the volume of the kidney tissue, collect the total protein solution, centrifuge, and then spot samples to denature the total protein solution. Prepare 10% separation gel and 5% concentrated gel, fill the gel immediately after adding TEMED, then start electrophoresis, transfer, and block, and incubate the primary and secondary antibodies at 4bC overnight. Drop the freshly prepared ECL mixed solution onto the protein side of the membrane for luminescence detection. The film is scanned and archived, and the AlphaEaseFC software processing system analyzes the optical density value of the target zone.

### 2.11. Statistical Analysis

The experimental data were analyzed by IBM-SPSS 22.0 software. The measurement data were described in terms of mean ± SD (*x* ± *s*). Each group was compared with analysis of variance (ANOVA), followed by independent t-test and Bonferroni posttest. Kruskal-Wallis analysis of variance was employed to determine the statistical differences of macro and micro scores among groups. *P* < 0.05 was considered to be statistically significant.

## 3. Result

### 3.1. Successfully Constructing an FD Rat Model with High Visceral Sensitivity

The period of intragastric administration of IA (13–20 days old) was marked by a significantly lower growth rate of body weight in the model group than that in the control group. At the age of seven weeks, no significant difference in body weight was documented among the other three groups. However, as illustrated in Figure 1(a), the body weight of rats in the model group was significantly lower than that in the control group at the age of seven weeks, one week after tail clamping stimulation (8 weeks old). The gastric sensitivity and compliance test results of eight-week-old rats witnessed no significant difference in electromyogram (EMG) RMS change rate and compliance of cervical trapezius muscle induced by gastric dilatation stimulation at 10–30 mmHg pressure between the control group and model group.  Figure 1(b) shows significantly higher root mean square change rate of the cervical trapezius muscle, whereas there was a significantly decreased gastric compliance in the model group compared with the control group, when the intragastric balloon pressure was 40–60 mmHg. No pathological alterations such as ulcers and bleeding were evident in the intestinal mucosa of the stomach and duodenum in all groups. As observed under the optical microscope, the intestinal mucosa of the stomach and duodenum in the model, EA, antagonist, and EA + antagonist groups were disordered, the intrinsic glands were relaxed, and a small amount of eosinophil infiltration was noted (which might be related to intestinal mucosal damage during visceral sensitivity measurement). The gastric and duodenal mucosal layers of rats in the control group were neatly arranged. There was no abnormality in the intrinsic glands. The structure of the submucosa and muscle layer was prominent with no obvious eosinophil infiltration (Figure 1(c)).

### 3.2. EA Mediates the Beneficial Effects of Visceral Hypersensitive FD

EA significantly enhances gastrointestinal motility. Compared with the control group, the gastric residual rate was increased, and the intestinal propulsion rate was significantly decreased in the other four groups. The previously mentioned results confirmed the successful establishment of the FD rat model in this experiment. Compared with the EA group, the gastric residual rate increased in the antagonist and EA + antagonist groups. Furthermore, a decrease in the intestinal propulsion rate was documented in the antagonist group and the EA + antagonist group compared with that of the EA group (Figure 2(a)).

EA reduces the number of mast cells in the duodenum and inhibits the activation and degranulation of mast cells. TB staining substantiated an increased number of mast cells in the other four groups compared with the control group. Nonetheless, the number of mast cells in the EA group, antagonist group, and EA + antagonist group decreased compared with the model group. Moreover, the number of mast cells in the EA group was lower than that in the antagonist group and EA + antagonist group. As seen in TEM, the morphology of mast cells in the control group was regular and quasi-round, and the cell membrane was intact and without degranulation. Compared with the control group, an irregularity was evident in the shape of mast cells in the model group, and there were many flocs around the cells, which were in the state of degranulation. However, with respect to the model group, the mast cells in the EA group were regular and oval, with few pieces of flocs around them, and the degree of degranulation was not obvious. Moreover, the morphology of mast cells in the antagonist group and EA + antagonist group was regular and oval, and there were few flocs around them. The degree of degranulation was not obvious (Figures 2 (b) and 2(c)). The results validated EA-induced significant activation and degranulation of mast cells in duodenal mucosa of VH in FD rats. Findings also confirmed that EA inhibited the number and activated degranulation of mast cells in duodenal mucosa.

### 3.3. EA Downregulates the Positive Expression of TRY, PAR2, PKC, and TRPV1 in Duodenal Mast Cells

The results from the experiments (Figure 3(a)) reflected an increased IOD value of TRY in the other four groups compared with the control group. However, the IOD value of TRY in the EA group, antagonist group, and EA + antagonist group decreased with regards to the model group. Furthermore, the IOD value of TRY in the EA group was lower than that in the antagonist group and EA + antagonist group. These findings revealed a significant increase in the release of TRY in the model group, whereas EA inhibited the release of TRY in duodenal mast cells.

EA reduces the expression of PAR2, PKC, and TRPV1 in the duodenum. As evident from Figure 3(b), enhanced IOD values of PAR2, PKC, and TRPV1 in the other four groups were manifested compared with the control group. On the other hand, the IOD values of PAR2, PKC, and TRPV1 in the EA group, antagonist group, and EA + antagonist group decreased compared with the model group. The IOD values of PAR2, PKC, and TRPV1 in the EA group were lower than those in the antagonist and EA + antagonist groups. Figure 3(c) confirms the previously mentioned results. Thus, the results confirmed significantly increased expression of PAR2, PKC, and TRPV1 in the model group and EA-mediated inhibition of the expression of PAR2, PKC, and TRPV1 in duodenal mast cells.

### 3.4. EA Diminished the Levels of PAR2, PKC, TRPV1, CGRP, and SP in DRG and c-fos in the Spinal Cord

Compared with the control group, increased IOD values for PAR2, PKC, and TRPV1 in the other four groups were obtained. Decreased IOD values of PAR2, PKC, and TRPV1 in the EA group, antagonist group, and EA + antagonist group compared with the model group. The IOD values of PAR2, PKC, and TRPV1 in the EA group were lower than those in the antagonist and EA + antagonist groups (Figure 4(a)). Overall, it was found that the expression of PAR2, PKC, and TRPV1 increased significantly in the model group, whereas EA inhibited the expression of PAR2, PKC, and TRPV1 in DRG.

EA reduces the expression of CGRP and SP in DRG. Increased IOD values of CGRP and SP in the other four groups were observed compared with the control group. A similar decrease in the IOD values of CGRP and SP in the EA group, antagonist group, and EA + antagonist group were observed concerning the model group. The IOD values of CGRP and SP in the EA group were lower than those in the antagonist group and EA + antagonist group. Figure 4(a) illustrates these findings. The results substantiated a significant increase in the expression of CGRP and SP in the model group, whereas EA impeded the expression of CGRP and SP in DRG.  Figure 4(b) also confirms that EA reduced the protein expression levels of PAR2, PKC, TRPV1, pTRPV1, CGRP, and SP in DRG.

EA reduces the expression of c-fos in the spinal cord. Compared with the control group, the IOD value of c-fos in the model group increased, while the IOD value of c-fos in the EA group, antagonist group, and EA + antagonist group was lower than that of the model group. Decreased IOD value of c-fos in the EA group was also witnessed than that in the antagonist group and EA + antagonist group (Figure 4(a)).  Figure 4(c) confirms that EA reduces the protein expression of c-fos in the spinal cord. These findings confirmed that EA repressed the expression of c-fos in the spinal cord.

Compared with the antagonist and EA + antagonist group, ^△^*P* < 0.05. Scale bar: 50 um.

## 4. Discussion

Early inflammatory stimulation is a predisposing factor for the formation of VH. The pathological mechanism of VH was better induced by the intragastric administration of IA as an early inflammatory response [20]. Anxiety and depression also repressed the visceral sensory threshold, enhancing the VH of patients [21]. In summary, our results well replicated the three pathological mechanisms of VH in FD, visceral hypersensitivity, decreased gastric compliance, and delayed gastric emptying. At present, the duodenum is believed to be the key site of functional gastroenteropathy symptoms [22, 23]. FD patients manifest a correlation between duodenal mast cells and neuronal signal changes. However, the potential disease mechanism of central sensitization has not been explored systematically [24]. Medium and small neurons in DRG are major targets for visceral pain signal transduction and regulation [25].

Studies have revealed that mast cell activation induces alteration in duodenal permeability and sensitivity in patients suffering from FD [26–28]. A positive correlation was noted between the symptoms of FD patients with the percentage of degranulated mast cells. FD patients demonstrated increased density and activity of mast cells in duodenal mucosa. Moreover, the expression of specific receptor TRPV1 targeting primary afferent nerve endings in duodenal mucosa increased significantly [29]. PAR2 receptor antagonists block visceral nociceptive sensory information, significantly improve acute and chronic colitis, reduce the activation and degranulation of mast cells, diminish the release of TRY, and alleviate VH [30]. In this study, the active site of mast cells in FD was expanded from the stomach to the duodenum. EA significantly decreased the number of mast cells in the duodenum, inhibited the activation and degranulation of mast cells, and downregulated the positive expression of TRY in duodenal mast cells.

PAR2 is one of the upstream molecules of PKC. Inhibition of PAR2 also impedes the activation of PKC [31, 32]. The role of the PAR2-PKC pathway in the generation and maintenance of pain has been well established [33]. The vital role of PKC, on the peripheral sensory nerve, especially PKC *ε*, is also observed in hyperalgesia caused by inflammation. The mechanism involves TRPV1 phosphorylation-mediated reduction of the open threshold of ion channels [34]. PKC *ε* activator aggravated the response of TRPV1 to capsaicin and temperature, while TRPV1 knockout mice failed to develop hyperalgesia when treated with PKC *ε* activator [35]. Meanwhile, PKC blocker induced alleviation of VH caused by TRY [36]. Our study found that the positive IOD values of PAR2, PKC, and TRPV1 in duodenum and DRG decreased following EA and with or without inhibitor treatment. The present study also revealed that the IOD values of PAR2, PKC, and TRPV1 in the EA group were lower than those in the antagonist group and EA + antagonist group. It is presumed that the expression of PAR2, PKC, and TRPV1 in the peripheral and central nervous systems was downregulated by EA.

Activation of TRPV1 on sensory neurons results in depolarization of neuronal cell membrane, directly or indirectly triggering afferent nerve endings to release sensory neuropeptides such as SP and CGRP and inducing VH [37, 38]. Alteration of visceral sensitivity is attributed to both central and peripheral CGRP release [39–41]. In the process of pain conduction in the spinal cord, neuropeptides, such as CGRP and SP, released at the central end of the primary afferent nerve fibers, contribute to the depolarization of neurons in the superficial layer of the posterior foot of the spinal cord [42]. The increased expression of c-fos during pain reflects the partial adaptive response of the spinal cord to continuous and subsequent nociceptive inputs [43, 44]. Our study highlighted EA-mediated significant reduction of the positive IOD values of neuropeptides CGRP and SP in DRG and c-fos in the spinal cord. EA also inhibited the expression of c-fos in the spinal cord induced by pain injury and effectively alleviated VH in FD rats.

There is growing evidence regarding the application of EA in relieving FD with VH. EA ameliorated gastric hypersensitivity in IA rats, which may be related to improving the balance of the sympathetic nerve and reducing the level of stress hormone [45]. Stress-induced gastric hypersensitivity in FD rats was blocked by adrenoceptor antagonists [46]. EA prevented or inhibited stress-induced gastric hypersensitivity by restoring sympathetic balance. To summarize, our results illustrated that EA and antagonists and EA + antagonists increased gastrointestinal motility and decreased the expression of PAR2, PKC, TRPV1, CGRP, SP, and c-fos downstream of PAR2/PKC pathway in FD rats, thus alleviating VH, though no significant superposition effect between antagonists and EA + antagonists was documented. Overall, our results strongly corroborated that EA regulates TRPV1 through PAR2/PKC pathway to improve VH in FD rats, and its protective mechanism is the comprehensive effect of multipathway and multitarget.

## Figures and Tables

**Figure 1:** Decrease in the growth rate of body weight and increase in the sensitivity in the model group. (a) The body weight in two groups at different times. (b) Stomach sensitivity and compliance. (c) HE staining of gastrointestinal tissue (× 200 magnification). No pathological alterations, including ulcer and bleeding, were observed in the intestinal mucosa of the stomach and duodenum in all groups. Scale bar: 100 um. Compared with the control group, ^※^*P* < 0.05, ^□^*P* < 0.0, ^#^*P* < 0.001, and ^△^*P* < 0.0001.

**Figure 2:** Electroacupuncture mediates the beneficial effects of visceral hypersensitive FD. (a) EA-mediated reduction in the residual rate in the stomach and increase in the propulsive rate of the small intestine in rats. (b) EA reduced the number and activation of mast cells in the duodenum. (c) The ultrastructural characteristics of fragmented or allergic degranulation of duodenal mast cells were observed under TEM (× 1700 magnification). Compared with the control group, ^△^*P* < 0.0001, ^□^*P* < 0.01; compared with the model group, ^#^*P* < 0.001, ^☆^*P* < 0.0001; compared with the EA group, ^※^*P* < 0.05, ^□^*P* < 0.01. Scale bar: 50 um.

**Figure 3:** EA downregulates the positive expression of TRY, PAR2, PKC, and TRPV1 in duodenal mast cells. (a) The positive expression of TRY in the duodenum was detected by immunohistochemistry (× 400 magnification). (b) The positive expressions of PAR2, PKC, and TRPV1 in the duodenum were identified by immunofluorescence (× 400 magnifications). (c) The protein expression levels of PAR2, PKC, TRPV1, and pTRPV1 in the duodenum were detected by western blot. Compared with the control group, ^△^*P* < 0.0001, ^□^*P* < 0.01; compared with the model group, ^☆^*P* < 0.0001; compared with EA group, ^※^*P* < 0.05. Scale bar: 50 um.

**Figure 4:** EA reduced the positive expression of PAR2, PKC, TRPV1, CGRP, and SP in DRG and c-fos in the spinal cord. (a) The positive expressions of PAR2, PKC, and TRPV1 in DRG were detected by immunofluorescence (× 400 magnification). (b) The protein expressions of PAR2, PKC, TRPV1, ptrpv1, CGRP, and SP in DRG were detected by western blot. (c) The protein expression of c-fos in spinal cord were detected by western blot. Compared with the control group, ^*∗*^*P* < 0.05, ^□^*P* < 0.01; compared with model group, ^#^*P* < 0.05, ^☆^*P* < 0.0001; compared with EA group, ^※^*P* < 0.05.

## Data Availability

The data used to support the findings of this study are available from the corresponding author upon request.
